# Development of a Clinical Prognostic Model for Metabolism-Related Genes in Squamous Lung Cancer and Correlation Analysis of Immune Microenvironment

**DOI:** 10.1155/2022/6962056

**Published:** 2022-09-06

**Authors:** Zifan Zhuang, Chundi Gao

**Affiliations:** ^1^College of First Clinical Medicine, Beijing University of Chinese Medicine, Beijing 100020, China; ^2^College of First Clinical Medicine, Shandong University of Traditional Chinese Medicine, Jinan, 250014 Shandong, China

## Abstract

**Background:**

The incidence of squamous lung cancer (LUSC) has substantially increased. Systematic studies of metabolic genomic patterns are fundamental for the treatment and prediction of LUSC. Because cancer metabolism and immune cell metabolism have been studied in depth, metabolism and the state and function of immune cells have become key factors in tumor development. This also indicates that metabolic genes and the tumor immune microenvironment (TME) are crucial in tumor treatment. This study is aimed at dissecting the connection between TME and LUSC digestion-related qualities.

**Methods:**

The information used in this study was obtained from The Cancer Genome Atlas dataset. Metabolism-related genes in patients with LUSC were screened, and relevant clinical data were collated. Next, genes associated with prognosis were screened using univariate COX regression and LASSO regression analyses. Finally, a timer database study was conducted to analyze the molecular mechanisms of immune cell infiltration of LUSC prognosis-related metabolic genes at the immune cell level.

**Results:**

Nine metabolism-related genes were identified: *ADCY7*, *ALDH3B1*, *CHIA*, *CYP2C18*, *ENTPD6*, *GGCT*, *HPRT1*, *PLA2G1B*, and *PTGIS*. A clinical prediction model for LUSC based on metabolism-related genes was constructed. In addition, 22 subpopulations of tumor-infiltrating immune cells (TIIC) in the TME were analyzed using the CIBERSORT algorithm. Finally, we used the TIMER database to analyze the immune infiltration of LUSC and the relationship between metabolism-related genes and immune cells.

**Conclusion:**

Our study identified metabolic genes associated with the prognosis of LUSC, which are important markers for its diagnosis, clinically relevant assessments, and prognosis. The relationship between metabolic genes with prognostic impact and immune infiltration was also analyzed, and a metabolic gene-based clinical prediction model was identified, providing a new perspective for LUSC treatment.

## 1. Introduction

Metabolism alludes to methodical compound responses that occur in an organic entity to support life. Cellular metabolism is crucial for cell survival and development. The first relationship between cancer cells and metabolism was demonstrated by Otto Warburg. He discovered that cancer cells would develop an abnormal dependence on glycolysis in the presence of sufficient oxygen. This phenomenon was called the “Warburg effect,” used to describe this particular form of aerobic glycolysis [1]. Different cancers exhibit different metabolic phenotypes. Generally accepted is that lactate contributes more to the tricarboxylic acid cycle than glucose in the metabolism of lung neoplasms [2]. There are many metabolism-related studies on different cancers, and they provide new ideas for studying tumor cell proliferation and patient survival. These metabolism-related processes are important because of the differences between the intrinsic signaling pathways within cancer cells and the interactions between cancer cells and their surrounding tumor immune microenvironment (TME) [3]. Accordingly, adjusting the digestion of cancer cells and upgrading the movement of insusceptible cells are significant challenges in the treatment of tumors.

We integrated the obtained clinical information with metabolism-related gene expression profiles to assess the prognostic status of patients with lung squamous carcinoma (LUSC). We systematically analyzed the prognosis of patients with LUSC and the expression of relevant metabolic genes. We identified key genes that can significantly affect patient outcomes and developed a new clinical prognostic model based on these genes. Immune infiltration associated with these genes was also analyzed. Our study provides a good basis for the treatment of LUSC in terms of metabolism and TME.

## 2. Methods and Materials

### 2.1. Data Assortment and Handling

Data related to patients with LUSC were obtained from The Cancer Genome Atlas (TCGA) (https://cancergenome.nih.gov/) and the corresponding clinical data [4]. All data required for this study were imported from the TCGA data download window GDC (https://portal.gdc.cancer.gov/), an open-access database from which the relevant information retrieved does not require additional moral approval. Only patients who were diagnosed with LUSC were included in this study. 504 tumor samples and 59 normal samples were obtained in total. Information on patients whose age and TNM stage were not recorded in the clinical data was also excluded from the relevant analysis. Finally, 494 tumor sample were obtained.

The Molecular Signature Database (MSigDB) is a set of annotated genomes that can be used in conjunction with centralized genome analysis software (https://www.gsea-msigdb.org/gsea/downloads.jsp). The background pathway gene set was downloaded from the website. Calibration to the same level and logfc of expression was performed by transforming the data using the R package. Metabolic-related genes were listed in the Kyoto Encyclopedia of Genomes (KEGG) according to the metabolic-related pathways in the Molecular Characterization Database [5].

### 2.2. Differential Expression Analysis and Pathway Enrichment Analysis

The expression data of metabolism-related genes in LUSC and normal lung tissues were normalized using the limma package in R software, and differential analysis was performed to obtain differential expression data of metabolism-related genes in LUSC in the TCGA database. The limit was set to absolute value of log2 (folding rate) > 1 and false discovery rate (FDR) < 0.05.

### 2.3. Risk Score Validation

To identify the genes most strongly associated with survival, we combined the expression of metabolism-associated genes with the OS of patients and then performed a univariate COX analysis on the sequential variables of genes. One-step screening further identified them as independent metabolic factors for predicting the prognosis of squamous lung cancer.

The screened metabolism-related genes were consolidated into Lasso regressions and repeated 1000 times using the glmnet package of R studio.

Last, a clinical prognostic model for LUSC was developed based on the LASSO regression coefficients multiplied by the expression figures. The equation is shown in the following equation.

(1) $$\begin{array}{c} \text{Risk}\cdot \text{score}=\alpha \text{gene}\left(a\right)\times \text{gene}\cdot \text{expression}\left(a\right)+\alpha \text{gene}\left(b\right)\times \text{gene}\cdot \text{expression}\left(b\right)+\cdots +\alpha \text{gene}\left(n\right)\times \text{gene}\cdot \text{expression}\left(n\right). \end{array}$$

### 2.4. Survival Analysis

Using the middle challenge score as the basic worth, we isolated patients with LUSC into generally safe gatherings and high gamble bunches. Kaplan–Meier curves were applied using the Survminer package of R to examine the association between metabolism-related genes and prognosis. Univariate and multivariate analyses were performed to investigate the free prognostic variables in patients with LUSC. The area under the curve (AUC) was determined using the endurance ROC R studio to confirm the prognostic highlights. Additionally, a nomenclature chart with clinical factors and chance scores was created. Calibration and decision curves were plotted to illustrate the accuracy of the model in predicting the survival of patients with LUSC.

### 2.5. GSEA

The purpose of the GSEA was to identify the pathways and molecular mechanisms (https://www.gsea-msigdb.org/gsea/index.jsp) associated with high- and low-risk groups. After 1000 substitutions, the gene sets with *P* < 0.05 and FDR < 0.05 were considered significantly enriched.

### 2.6. Analysis of the Relationship between Immune Cell Infiltration and Metabolism-Related Genes

Investigations have shown that metabolism and TME play a significant role in cancer treatment. The highly active metabolic pathways peculiar to cancer cells can profoundly change the components of many small molecules, as well as the nutritional products in the TME. The high metabolic activity and unorganized blood vessels of cancer cells in the TME contribute to nutrient depletion and hypoxia, leading to a metabolic contest between cancer cells and invading invulnerable cells [6–8]. All immune-related data for LUSC were obtained from the TCGA and transformed into TPM matrices using the R software preprocess core package to obtain immune cell content, the estimation package to obtain the TME scores, and the corrplot package for immune-related analysis. And based on this data, the proportion of 22 immune cells in LUSC was plotted. The TIMER database (https://cistrome.shinyapps.io/timer/) was used to analyze and visualize the number of tumor-infiltrating immune cells and examine the correlation between metabolism-related genes screened by LASSO regression and the level of infiltration of six immune cell subtypes: CD4+ T cells, B cells, CD8+ T cells, neutrophils, macrophages, and dendritic cells. Copy number variation is an important aberration that leads to changes in gene expression during tumorigenesis and cancer growth. TIMER applied data from GISTIC 2.0 to examine the impact of genes with different copy states on immune infiltration, including CD4+ T cells, B cells, CD8+ T cells, neutrophils, macrophages, and dendritic cells.

## 3. Result

### 3.1. Screening of Metabolism-Related Genes

Gene expression analysis was performed on 504 and 59 tumor and normal specimens, respectively. Among them, there were 504 tumor samples, and 494 samples remained after their exclusion due to partial lack of data such as survival time. We identified metabolic-related genes from the KEGG genome (Supplement 1). Among the genes screened for differential expression based on profiles, 353 were upregulated, and 197 were downregulated in tumor specimens (*P* < 0.05, Figure 1(a)). For additional determination, 14 genes proved to be of prognostic significance based on the calculated HR values of patients with LUSC by univariate COX regression analysis. Eleven of these genes (*ADCY7*, *ALDH3B1*, *ALOX5*, *AOC3*, *CHIA*, *ENTPD6*, *PDE2A*, *PLA2G15*, *PLA2G1B*, *PTGIS*, and *SGMS2*) may have more terrible anticipation than the other three genes (*P* < 0.01, Figure 1(b)).

### 3.2. Developing the Expectation Model

As aforementioned, we identified candidate metabolic genes associated with prognosis. For the selected genes, we performed LASSO regression to build the model and determine the coefficients. Finally, the model contained nine genes, with every coefficient mathematically showing the heaviness of articulation. Individual risk scores were determined based on the articulation status of prognostic qualities and their related coefficients (*P* < 0.05, Table 1).

The calculation formula of the risk score was shown as the following equation:

(2) $$\begin{array}{c} \text{Risk}\cdot \text{score}=\left[\begin{array}{c} \text{ADCY}7*\left(0.0396025207343667\right)+\text{ALDH}3\text{B}1*\left(0.011687487660189\right)\\ +\text{CHIA}*\left(0.0143573936898486\right)+\text{CYP}2\text{C}18*\left(-0.0356322600211849\right)\\ +\text{ENTPD}6*\left(0.0196686829383862\right)+\text{GGCT}*\left(-0.00384755414754328\right)\\ +\text{HPRT}1*\left(-0.00251832392113586\right)+\text{PLA}2\text{G}1\text{B}*\left(0.0193309813261464\right)\\ +\text{PTGIS}*\left(0.027941353204922\right) \end{array}\right]. \end{array}$$

### 3.3. Confirmation of Risk Scores

To further affirm the reliability of the risk scores, we divided the TCGA LUSC cohort into two groups based on their median risk scores: high- and low-risk. Analysis of the pathways involved in the high- and low-risk groups by using the GSEA predictions showed that the risk scores were significantly enriched in several metabolically related bioprocesses (Figure 2(a)). It can be clearly seen that the enrichment of genes in metabolism-related and other pathways is significantly different between the high-risk and low-risk groups. In the high-risk group, 119 gene sets are upregulated, and 104 gene sets are significant at FDR < 0.25. In the low-risk group, 59 gene sets are upregulated, and 31 gene sets are significant at FDR < 0.25. K-M survival analysis showed that survival probability in the low-risk group was much higher than in the high-risk group (Figure 2(b)).

The distribution of the risk scores and the correlation between survival data are shown in a scatter plot (Figure 3(a)). Based on the value of the median risk score in the TCGA LUSC cohort, patients were separated into low- and high-risk groups (Figure 3(b)). The expression profiles of prognostic risk genes between the high- and low-risk groups are shown in the heat map (Figure 3(c)).

### 3.4. Analysis of the Combination of the Risk Scoring System and Clinical Factors

Based on the analysis of univariate and multivariate LASSO Cox regression models, we found that a risk scoring system constructed using mRNA could be used to predict OS in patients with LUSC. To further evaluate its predictive performance, we constructed ROC curves. This implies that the risk scoring system has an excellent predictive ability (Figure 4(c)). Univariate Cox analysis showed that stage, T-stage, and risk score were significantly associated with OS (Figure 4(a)). Further multivariate Cox analysis revealed that risk score could be used as independent prognostic factors to assess patient survival time (Figure 4(b)). Regardless of the univariate or multivariate analyses, the risk score system we constructed was very effective in assessing the prediction, which further showed the assessment value of the model.

### 3.5. Metabolic Genes and the Immune Microenvironment

The proportion of the 22 immune cells in LUSC is shown in Figure 5. Pearson correlation analysis illustrates the coexpression pattern between immune cells with a significant positive correlation between CD4 memory-activated T cells and CD8 T cells and a negative correlation between CD8 T cells and macrophages M0 (Figure 5).

To understand whether the metabolic genes used to construct the prognostic model were associated with the immune microenvironment, the association between nine genes of prognostic significance (*ADCY7*, *ALDH3B1*, *CHIA*, *CYP2C18*, *ENTPD6*, *GGCT*, *HPRT1*, *PLA2G1B*, and *PTGIS*) and immune infiltration was analyzed using the TIMER database. As shown in Figure 6, the expression of six genes, *ALDH3B1*, *CHIA*, *GGCT*, *HPRT1*, *PLA2G1B*, and *PTGIS*, correlated significantly (*P* < 0.05) with immune infiltration in all six cell types; the expression of *ADCY7* and *CYP2C18* correlated with CD4+ T cells, CD8+ T cells, neutrophils, macrophages, and dendritic cells (*P* < 0.05), and the expression of *ENTPD6* correlated significantly with the infiltration of B cells and CD8+ T cells (*P* < 0.05). In addition, we analyzed the relationship between somatic copy number changes and the abundance of the immune infiltration of metabolism-related genes (Figure 7). The SCNA module provides a comparison of the level of tumor infiltration for a given gene with different somatic copy number changes. SCNA is defined by GISTIC 2.0 and includes deep deletion, arm-level deletion, diploid/normal, arm-level deletion, and high amplification. Box plots show the distribution of each immune subset at each replicate number state in the LUSC.

## 4. Discussion

Metabolism is a critical aspect in the development of cancer, and tumor tissues tend to exhibit faster metabolic capabilities, such as glucose metabolism, than normal tissues, to fulfill their rapid growth. It also affects the protocol and efficacy of tumor immunotherapy. The study of tumors must continue. Research at the genetic level is expanding, and differentially expressed genes play an important role in cancer research and subsequent related therapies. We thoroughly investigated the impact of metabolic genes on the prognosis of LUSC and elaborated on the related mechanisms by selecting 14 closely related genes. Using these genes, we assessed the clinical features associated with LUSC.

From the 14 metabolic genes obtained, we screened 9 genes (*ADCY7*, *ALDH3B1*, *CHIA*, *CYP2C18*, *ENTPD6*, *GGCT*, *HPRT1*, *PLA2G1B*, and *PTGIS*) using LASSO regression. Based on these nine genes, a correlation model was developed to understand tumor metabolism in patients, predict disease outcomes, and guide clinical treatment. We combined the models and found that the low-risk group tended to show longer survival times than the high-risk group, and the reliability of the models was confirmed by regression analysis. Our study suggests that clinical prognostic models using metabolic genes can be used as indicators for an independent analysis.

The expression level of ADCY7 affects several human metabolic processes and affects many important physiological aspects of the body, especially with a strong correlation with the level of immune cell infiltration. The literature has demonstrated that ADCY7 and the prognosis of acute myeloid leukemia are closely related, and its high expression may be detrimental to the prognosis of patients with this disease [9]. Studies have confirmed that *ALDH3B1* is expressed at higher levels in lung adenocarcinoma tissues than in normal tissues. This expression has an important impact on the prognosis of other cancers such as lung adenocarcinoma. A commonly held belief is that the expression of *ALDH31* affects the metabolism of aldehydes such as acetaldehyde [10]. Aldehydes have stimulatory effects in humans and induce mutations that lead to cancer [11]. Studies have confirmed that *ALDH3B11* is relatively highly expressed in mouse lung tissue, where it plays an important role in aldehyde metabolism. This mutation is likely to cause lung lesions [12]. *GGCT* is also involved in important metabolic processes in the body, catalyzing the production of 5-oxoproline and free amino acids [13, 14], and the literature has shown that *GGCT* expression is upregulated in clinical samples from various cancers. Studies have identified elevated *GGCT* expression in 58% of cervical cancers, 38% of lung cancers, and 72% of colon cancers [15]. *GGCT* inhibitors are currently used as anticancer drugs.

Undoubtedly, attempts to understand the mechanism of tumorigenesis have increased in sophistication and comprehensiveness. However, many questions remain even though an inextricable link between metabolism and cancer has been identified. For LUSC, many aspects of the relevant mechanisms remain unclear. Our study focused on the link between the tumor metabolic state and the immune environment.

Accelerated tumor growth is a major explanation for the inability of immune cells to monitor and eliminate it on time [16]. Tumor cells may evade the body's immune surveillance under the influence of various factors, such as by downregulating the expression of relevant antigens; however, some tumor cells are inherently weakly immunogenic or release soluble antigenic factors to close off receptors [17]. Studies have shown that nonsmall cell carcinomas can establish multiple immune escape mechanisms [18]. Tumor cells upregulate the glycolytic catabolism of glucose to form lactate, which also induces the formation of an immunosuppressive environment, and its concentration is also influenced by macrophages [19].

Cancer cells depend on glucose and lipid uptake for survival and growth, and the TME often reflects the immune status of cancer cells and can provide strong support for subsequent therapeutic strategies. Different members of the TME, which constitute the specific ecological environment of the tumor, interact through cytokines, chemokines, and other factors. A necessary linkage has been made between TME and metabolic gene correlation. Additionally, metabolism-related genes, such as those affecting glycolysis, have been shown to play an important role in the proliferation and invasion of cancer cells.

First, we demonstrated the feasibility of constructing a model based on nine metabolism-related genes to determine the clinical treatment of LUSC. Cancer development is closely related to metabolism; however, immunity plays a more critical role than metabolism. Cellular metabolism is the key to maintaining the viability and function of cancer and immune cells. Immunotherapy is an established tool for cancer treatment [20]. By analyzing the data obtained using the ESTIMATE algorithm, we obtained immune and matrix scores to understand the LUSC microenvironment. Next, we used CIBERSORT to assess the different infiltration patterns of various immune cells in patients with LUAD and LUSC and reveal their relationship with clinical outcomes. Most TIICs in LUSC were significantly different from those in normal tissues, suggesting a critical role of immune status in cancer progression, and there is a clear coexpression pattern between some related immune cells. Recent research has found that the content of neutrophil infiltration in tumor tissue was significantly altered in LUSC [21, 22].

We also found that the expression of genes related to metabolism was associated with the degree of infiltration of immune cells, such as CD4+ and CD8+ T cells. The literature has shown that most of the follicular B cells infiltrated by tumors are highly expressed to CD40 and so forth [23]. Plasma cells are thought to be associated with better long-term survival in NSCLC, suggesting an active role for plasma cells in antitumor immunity [23, 24]. Tumor-infiltrating lymphocytes (TIL-Bs) play a regulatory role in activating B cells but can also influence the density of T cells [25]. T cells play an important role in immune processes and are a central component of tumor cell immunity. CD4+ T cells express various costimulatory molecules that can be activated by interactions with other immune cells, such as B cells [26, 27]. CD4+ T cells belong to the family of tumor necrosis factor receptor costimulatory receptors and are associated with NSCLC tumor frequency [28]. Additionally, CD8 T cell-derived metabolites can mediate fatty acid metabolism through blockade [29].

In conclusion, T cell metabolites have an important impact on antitumor immune responses. Tumor-associated macrophages are the major immune-infiltrating cells in the TME [30–32]. Relevant studies have shown that their metabolites contribute to tumor invasion and metastasis, and metabolite analysis may improve the understanding of the hyperprogressivity of cancer in immunotherapy [33].

This study has limitations. First, we had limited access to data information, which reflected only part of the tumor immunity and metabolism. Second, we did not include an independent cohort for validation. Finally, our results require validation through relevant experiments.

## 5. Conclusion

In summary, based on the relevant data downloaded from the TCGA database, a screening of metabolism-related genes associated with the prognosis of LUSC patients was performed. A prediction model was constructed based on nine metabolism-related genes (*ADCY7*, *ALDH3B1*, *CHIA*, *CYP2C18*, *ENTPD6*, *GGCT*, *HPRT1*, *PLA2G1B*, and *PTGIS*). The immune microenvironment was also analyzed based on metabolism-related genes, and the association between metabolism-related genes and immune cells was analyzed using the TIMER database. This study has guiding significance for LUSC prognosis, which benefits future in-depth exploration of immune- and metabolism-related mechanisms of LUSC.

## Figures and Tables

**Figure 1:** Selection of candidate genes. (a) Volcano plot of differential gene expression between tumor and normal tissues. Red dots represent upregulated genes. Green represents downregulated genes. Genes without significance are marked in black. (b) Genes significantly associated with prognosis after the secondary screening. Red and green dots represent the HR of the corresponding genes above and less than 1, respectively. FC: fold change; HR: hazard ratio.

**Figure 2:** GSEA and survival analysis. (a) Representative results of GSEA analysis of high- and low-risk group genes. (b) Survival curve for OS. The red line depicts the survival of high-risk patients; the blue line depicts the survival of low-risk patients.

**Figure 3:** Validate risk scores. (a) Distribution of risk scores for the high-risk and low-risk groups. Red dots indicate cases in the high-risk group, and green indicates low-risk cases. (b) Distribution of survival status of patients in the high-risk and low-risk groups. Green dots represent alive and red dots represent dead. (c) Heat map of the expression profiles of metabolism-related genes included.

**Figure 4:** Forest plots. For (a) univariate and (b) multivariate Cox regression analysis in the TCGA LUSC cohort. (c) ROC curves for risk scores. AUC: area under the curve.

**Figure 5:** Proportion of immune cells per patient. The blue and red graphs indicate a negative and positive correlation, respectively.

**Figure 6:** Correlation of metabolism-related genes and immune cell infiltration levels in human LUSC analyzed using TIMER database. (a) *ADCY7*, (b) *ALDH3B1*, (c) *CYP2C18*, (d) *ENTPD6*, (e) *GGCT*, (f) *HPRT1*, (g) *PLA2G1*, (h) *PTGIS*, and (i) *CHIA* levels were closely correlated with tumor immune cell infiltration in LUSC.

**Figure 7:** Correlation of somatic cell replication number alteration (SCAN) with the abundance of immune infiltration of neoplastic hypometabolism-related genes analyzed using the TIMER database. (a) *ADCY7*, (b) *ALDH3B1*, (c) *CHIA*, (d) *CYP2C18*, (e) *ENTPD6*, (f) *GGCT*, (g) *HPRT1*, (h) *PLA2G1*, and (i) *PTGIS* include deep deletion, arm-level deletion, diploid/normal, arm-level gain, and high amplification. The box plot shows the distribution of each TIIC subset for each copy number status in LUSC using the same statistical tests as the “Mutation” module.

**Table 1:** Characterization of LUSC metabolic genes and coefficient of risk.

Gene	Coef
ADCY7	0.0396025207343667
ALDH3B1	0.011687487660189
CHIA	0.0143573936898486
CYP2C18	-0.0356322600211849
ENTPD6	0.0196686829383862
GGCT	-0.00384755414754328
HPRT1	-0.00251832392113586
PLA2G1B	0.0193309813261464
PTGIS	0.027941353204922

## Data Availability

The data is public and can be downloaded from the TCGA database for free.

## Abbreviation

LUSC: Squamous lung cancer
TME: Tumor microenvironment
TIIC: Tumor-infiltrating immune cells
NSCLC: Nonsmall cell lung cancer
OS: Overall survival
FDR: False discovery rate
LASSO: Least absolute shrinkage and selection operator
AUC: Area under the curve
K-M: Kaplan-Meier.

## Supplementary Materials

Supplementary Materials Supplement 1: metabolism-related genes in lung squamous cell carcinoma.
